The article "Nursing Diagnosis of Urology Operating Room Based on New Association Classification Algorithm" was retracted in 2023. Reasons: signs of a paper mill; compromised peer review; unreliable results or conclusions.

# Nursing Diagnosis of Urology Operating Room Based on New Association Classification Algorithm

**DOI:** 10.1155/2022/4674959

**Published:** 2022-04-06

**Authors:** Hongyan Zhang

**Affiliations:** Urology Endoscopy Room, the First Affiliated Hospital of Harbin Medical University, Harbin, Heilongjiang 150001, China

## Abstract

Due to the rapid development of medical engineering, massive amounts of data are recorded and preserved by various medical instruments. Therefore, finding relationships among data and summarizing clinical manifestations are of great significance to the diagnosis, treatment, and medical research of various diseases. The key to studying the nursing diagnosis support system, particularly in the urological operating room, is to select an effective classification algorithm, which is suitable for the characteristics of urological diseases. Initially, we have analyzed characteristics of urological diseases through medical data mining. Secondly, based on the traditional data mining classification method and urological disease diagnosis research, we have introduced the urological disease experimental source dataset and analyzed characteristics of the disease. Furthermore, classification algorithm and steps were introduced such as decision tree (including ID3, C4.5), Bayesian classification, BP neural network, and association rule classification algorithms. These algorithms are used to make relevant comparative experiments on the urological disease dataset. Finally, based on the diagnosis of urological diseases, a new association classification algorithm (ACCF), which is based on frequent closed item sets, is proposed along with suitable explanation. In order to verify the operational capabilities, the proposed algorithms are implemented in *C*++ and compared with the classification effect of traditional association classification algorithms and data mining methods. Both theoretical analysis and experiment results show that the proposed algorithm has resolved various deficiencies of the existing data mining algorithms and equally improved the accuracy of urological disease classification and prediction.

## 1. Introduction

Generally, urinary surgery patients have different degrees of pain symptoms particularly after the surgery. Pain not only aggravates negative emotions but also equally reduces the degree of cooperation, compliance, and the body's recovery speed. However, due to the development of society and economy, people's material living standards have significantly improved and requirements for the quality of healthcare are also getting higher and higher. Traditional nursing methods are difficult to meet the current clinical and patient needs. It is easy for nurse-patient disputes to occur, but it has certain limitations. Comprehensive nursing intervention pays attention to all details of nursing service. Intraoperative heat preservation care for patients is strengthened, which effectively reduces the incidence of hypothermia and is safer. Comprehensive nursing intervention allows patients and their families to feel the responsibility and professionalism of the nursing staff. Trust the nursing staff more, shorten the distance between each other, build a harmonious and good doctor-patient relationship, and improve the quality of nursing service in the hospital.

The article "Nursing Diagnosis of Urology Operating Room Based on New Association Classification Algorithm" was retracted in 2023. Reasons: signs of a paper mill; compromised peer review; unreliable results or conclusions.

With the rapid development of computer technology, especially the widespread application of Internet-related technologies and database systems, massive amounts of data have been generated. These mass data have prompted people to put forward higher requirements for data analysis tools. Although the current database system can realize the functions of adding, querying, updating, and deleting data, it is difficult to discover the relationships and laws between the data. Faced with such challenges, in order to extract useful information and knowledge from massive data to guide people's practical activities in production and life, Data Mining Technology emerged at the historic moment. After more than 20 years of rapid development, it has become a kind of interdisciplinary subject, integrating related fields such as database, statistics, machine learning, artificial intelligence, and high-performance computing. Recent research studies mainly focus on classification, clustering, association rule mining, and forecasting and trend analysis. Thus, data mining technology, as the most effective means to solve the lack of information caused by data explosion, has received great attention from academia and business circles [1–3].

In recent years, medical engineering has developed rapidly, and a large amount of medical information has been recorded in detail, leading to a massive increase in medical data. Especially, with the widespread application of medical information systems in major hospitals, the recorded case data include a variety of physiological indicators, medical images (X-ray images, B-ultrasound images, color ultrasound images, etc.), as well as gender, height, detailed background information data such as weight, age, and previous medical history. The amount of data is very huge, and these are real case information. In such a huge dataset, data mining methods and techniques are used to discover and summarize the clinical manifestations of various diseases and the interrelationships between various diseases. The development law of the disease and the efficacy of various treatment programs are very valuable and meaningful for the diagnosis and treatment of the disease and even for medical research [4].

The article "Nursing Diagnosis of Urology Operating Room Based on New Association Classification Algorithm" was retracted in 2023. Reasons: signs of a paper mill; compromised peer review; unreliable results or conclusions.

In the current medical process, especially in the diagnosis and treatment, diagnosis of diseases by doctors is still in a relatively traditional experience stage, and the diagnosis results are largely determined by various diagnostic indicators and the doctor's own clinical practice experience. The lack of practical experience of clinicians will definitely lead to misjudgment of the final diagnosis [5]. In general, a clinician can accumulate relevant diagnostic experience through many years of actual diagnostic activities. If the diagnostic knowledge and experience that can be compared with experts in the field are discovered, they can be provided to the majority of medical staff in a more convenient way so as to reduce the subjective blindness of diagnosis to a large extent, making the diagnosis result more accurate, and further improve the diagnosis level of the disease [6, 7].

Under the background of our country's medical reform, it is an inevitable trend to actively seek to use information technology to advance the reform of the medical industry. The use of data-mining-related methods and technologies in the clinical decision support system of urology has the following significance:

1. Study application of data-mining-related methods and technologies in practice, and promote the research and development of related theories.
2. To study the characteristics of urological diseases, discover the clinical characteristics of the disease, formulate effective diagnosis and treatment methods, and provide clinical doctors in the field of urology with decision-making support in diagnosis and treatment such as the use of association rules of classification methods combined with urology theories. To study the relationship between the disease and the patient's gender, weight, diet, etc., to further discover the cause of disease and formulate a treatment plan.
3. Based on the mining of a large number of case data, certain rules can be found to provide decision-making support for the management.

To solve the existing issues, a nursing diagnosis of urology operating room (Figure 1) based on new associated classification is proposed in this paper. The major scientific contributions of this paper are given as follows:

- Thorough analysis of the characteristics of urological diseases through medical data mining.
- Introduction of the urological disease experimental source dataset, which is primarily based on traditional data mining classification and urological disease diagnosis methods.
- Classification algorithm and steps to make relevant comparative experiments on the urological disease dataset.
- Finally, based on the diagnosis of urological diseases, a new association classification algorithm (ACCF) is proposed with maximum accuracy and precision ratio.

The article "Nursing Diagnosis of Urology Operating Room Based on New Association Classification Algorithm" was retracted in 2023. Reasons: signs of a paper mill; compromised peer review; unreliable results or conclusions.

The remaining manuscript is organized as given in the following paragraph.

In subsequent sections, a comprehensive and detailed review of the relevant literature is provided where existing state-of-the-art methods are described in detail along with identification of various issues.

## 2. Related Work

The rapid development of computer technology has led to the rapid development of artificial intelligence and knowledge engineering. Expert systems is the branch with the most extensive applications and the most obvious achievements [8]. It is a computer system with rich professional knowledge and experience. It uses artificial intelligence and computer-related technologies to perform deduction and discrimination based on information provided by several experts in the industry, and it simulates the decision-making process of human experts to deal with those needs. Complex issues dealt with by human experts. Now expert systems have been widely used in many fields such as engineering, science, medical treatment, military, and commerce, and have achieved fruitful results [9].

Medical expert system is the use of computer technology to replace medical experts to process those clinical medical data, combined with the design principles and methods of expert systems, to simulate the process of synthesis, analysis, diagnosis, and treatment of diseases by medical experts. It can be used to help doctors solve a variety of medical problems, as an auxiliary tool for doctors' diagnosis, treatment, and prevention [10], which can also save, organize, and disseminate important theories and a large amount of clinical practice experience of medical experts. Among these methods, the most widely used method is the decision support system that helps doctors make clinical diagnosis decisions [11]; therefore, the medical expert system is also called the clinical decision support system (CDSS).

In 1974, Short liffe and others, who belong to Stanford University in the United States, successfully developed the MYCIN system with high performance for the first time to help physicians diagnose and treat infectious diseases. Since then, a large number of clinical decision-making systems have emerged such as University of Pittsburgh. In 1982, Miller successfully developed the famous Internist-I internal medicine computer-aided diagnosis system [12]. Its knowledge base contains 572 types of diseases and about 4,500 symptoms. These are relatively large-scale clinical decision support systems. In addition, many people have successfully developed many special clinical decision support diagnosis systems for a certain disease or a certain type of disease. In 1990, Umbaugh developed auxiliary diagnosis system for skin cancer successfully [13]. A diagnostic decision support system for the diagnosis of chronic abdominal pain was developed by Provan in 1994 [14]. In 1996, Ling established a representative AIDS medical expert diagnostic system [15]. Wells successfully developed a diagnostic system in 200 years which is used to help treat breast cancer diseases [16]. The successful development and application of this large number of clinical decision support systems not only facilitates doctors and patients but also greatly promotes the research and development of medical science.

The article "Nursing Diagnosis of Urology Operating Room Based on New Association Classification Algorithm" was retracted in 2023. Reasons: signs of a paper mill; compromised peer review; unreliable results or conclusions.

The earliest clinical decision support system in our country was the “Guan Youbo Liver Disease Diagnosis and Treatment Program” developed by the famous professor Guan Youbo and others in the Beijing Hospital of Traditional Chinese Medicine in 1978. This system is based on the theory of Chinese medicine, and then China's clinical decision support system has the deepest development in Chinese medicine. Then, Jilin University and Bethune Medical University successfully developed the “Chinese Medicine Gynecology Expert System” [17]. Since then, various domestic industries have also successfully developed various clinical decision support expert systems for specific medical fields, such as the Chinese medicine expert System [18], the diagnosis system of coronary artery calcification points based on spiral CT images [19], the diagnosis of palm prints Expert System [20], Bone Tumor Aided Diagnosis Expert System [21], Ear Acupoint Information Intelligent Recognition System [22], duodenal ulcer diagnosis expert system [23], gastric cancer diagnosis expert system [24], etc. Among them, in 2003, Yi Tao and others developed a cardiovascular drug treatment expert system, which uses case-based reasoning to solve the problem of clinicians obtaining medication knowledge and experience.

At present, data-mining-related methods and technologies are widely used in clinical decision support systems, such as the application of Bayesian networks in the diagnosis of mild cognitive impairment, and the research and application of neural networks in the EEG signal diagnosis expert system, research and application of fuzzy clustering in intelligent medical diagnosis system, and so on. The establishment of these systems has greatly promoted the interdisciplinary research, but until today, there is still no clinical decision support system that can be widely used in clinical practice. To explore the reasons, we believe that the main problems are as follows:

The article "Nursing Diagnosis of Urology Operating Room Based on New Association Classification Algorithm" was retracted in 2023. Reasons: signs of a paper mill; compromised peer review; unreliable results or conclusions.

### 2.1. Current Clinical Decision Support System

The most extensive and deepest research in the current clinical decision support system is the disease diagnosis expert system, which is positioned to provide doctors with diagnosis tips for several common symptoms or diseases in practical applications, but this is hardly a problem for a doctor with actual clinical experience. This is because accurate diagnosis of diseases is very important to patients. Simple diseases are usually diagnosed by doctors, while complex diseases often require multiple doctors' consultations and even lengthy and repeated examinations. The disease evolves and diagnostic treatment can be implemented. Some systems are positioned for patients' self-diagnosis of diseases, but this positioning is not only difficult to promote; even if it can be promoted, it is only a software similar to health consultation, and it is harder to talk about broad application prospects.

### 2.2. Lack of Interdisciplinary Talents

The establishment and improvement of the clinical decision support system requires the input of a large amount of case knowledge and continuous learning, correction, and optimization in practical activities. The whole process requires relevant personnel to have a deep clinical medical diagnosis background. However, clinical medicine is a very professional subject. With its long learning cycle and busy daily work, it is difficult for clinicians to learn computer-related knowledge. However, the main relevant personnel of the clinical decision support diagnosis system are those with computer or biomedical engineering background, so it is likely to cause many defects in such a system.

### 2.3. Lack of Supervision of Doctors

Under the current medical system, the supervision of doctors is very important. This is because a few doctors with low medical ethics do not follow the medical guidelines due to the shortcomings of the current medical system. They have random inspections, random prescribing behaviors, and some medical skills. Inferior doctors can even cause medical accidents and so on.

## 3. Method

### 3.1. Research on the Diagnosis of Urological Based on Traditional Data Mining

Throughout the doctors' diagnosis process, we can find that the diagnosis process of a disease is the process of classifying the patient into a certain disease category according to the disease characteristics (sickness) of the patient. In fact, it is also a disease classification process. Therefore, the key to studying the clinical decision support system of urology is to choose an effective classification algorithm suitable for the characteristics of urology diseases.

The article "Nursing Diagnosis of Urology Operating Room Based on New Association Classification Algorithm" was retracted in 2023. Reasons: signs of a paper mill; compromised peer review; unreliable results or conclusions.

#### 3.1.1. Overview of Classification Algorithms

In data mining, classification is the most widely used and the most studied method. The classification method learns the difference of each category from the past classified empirical data, and establishes a model to describe the difference. It can be used to describe the data or classify the unknown category of data. The model is also called a classification function or classification model (also called classifier in general). The process of building a model is usually divided into two stages: training and testing. Before building a model, generally the dataset needs to be randomly divided into two parts: training dataset and test dataset. In the training phase, the training dataset is used to study the dataset samples described by the attributes to build the model. It is assumed that each sample belongs to a known class. The class is determined by an attribute called the class label. The form can be expressed as: (u1, u2, ... Un; c), where u1 represents the attribute value and *c* represents the category. The training phase is also called guided learning, because the class labels of the samples used in this phase have been determined. In general, the form of the model is expressed as a decision tree, classification rule, or mathematical formula. In the testing phase, the test dataset is used to evaluate the classification accuracy of the model. If the classification accuracy is deemed to have reached the measurement standard, then the classification model can be used to classify new data samples of unknown classification. Under normal circumstances, the cost of the training phase is much higher than that of the test phase, so the general data mining methods ignore the cost of the test phase.

Classification has been widely applied and researched in many fields. So far, the traditional classification methods that have been researched mainly include: decision tree methods (traditional decision tree classification algorithms mainly include ID3 algorithm, C4.5 algorithm, and so on), Bayesian classification, genetic algorithm, neural network method BP algorithm, K2 nearest neighbor algorithm, case-based reasoning, etc. Associative classification, support vector machine (SVM), rough set method, and fuzzy set method are the hot and newer methods that have been studied in recent years.

#### 3.1.2. Decision Tree Classification

Decision tree is one of the most widely used inductive deduction methods. It is based on examples and is generally used to build classifiers and predictive models. Its classification rules are represented by a decision tree, deduced from a set of disorderly and irregular cases. It uses a top-down recursive method to compare the attribute values at the internal nodes of the decision tree to classify the types. A path from the root to the leaf node corresponds to a conjunctive rule, and the entire decision tree corresponds to a set of disjunctive expression rules. To improve readability, the decision tree obtained by training is also expressed in the form of multiple if-then rules. Quinlan published the famous ID3 algorithm paper in 1986. Based on the ID3 algorithm, Quinlan published a paper on the C4.5 algorithm in 1993. Both algorithms, i.e., ID3 and C4.5, are briefly described here.

(a) ID3 Algorithm
    The key idea is that when selecting attributes at all levels of the decision tree, the selection criterion is information gain, so that when each nonleaf node is tested, the largest category of information about the tested sample can be obtained. The specific method is: (i) calculate all the attributes, (ii) select the attribute with the largest information gain as root node of the entire decision tree, (iii) construct different branches according to the value of node, (iv) and recursively call the previous process for each branch. The branch of the node is further constructed until all the subsets only contain the data of the same category label. In the end, a decision tree will be obtained, which is the final classifier, which can classify data samples of unknown classification.
    The theory of information gain method is derived from the principle of information entropy. Information entropy is used to measure the level of information confusion. Generally speaking, if the information is uniformly mixed and distributed, the information entropy is high. If the information is uniformly distributed, the information entropy is low. In the decision tree, “information” is represented by class labels, that is, if the categories in the data subset are mixed and evenly distributed, the information entropy is higher. If the category is uniformly distributed, the information entropy is low. By comparing the change of information entropy before and after the division of each attribute, and selecting the attribute that makes the information entropy change in the smallest direction, the decision tree can quickly reach the leaf nodes, so that a compact decision tree can be constructed.
    The advantages of ID3 algorithm are: simple method, clear theory, and strong learning and training ability. The disadvantage is that it is more sensitive to noise data and is only effective when the dataset is small.
(b) C4.5 Algorithm
    The C4.5 algorithm inherits the advantages of ID3 and improves the following aspects: The use of information gain rate as the criterion for attribute selection improves the shortcomings of bias in selecting attributes with more values when information gain is used as the criterion. The advantages of C4.5 are: the generated classification rules are simple and easy to understand, and the accuracy is high. The disadvantage is: in the process of building a decision tree, the dataset needs to be scanned and sorted many times, which makes C4.5 inefficient. Moreover, C4.5 stores all the datasets in the memory during the training process. When the training set exceeds the memory capacity, C4.5 will not be able to run.

The article "Nursing Diagnosis of Urology Operating Room Based on New Association Classification Algorithm" was retracted in 2023. Reasons: signs of a paper mill; compromised peer review; unreliable results or conclusions.

#### 3.1.3. Bayesian Classification

Bayesian classification is a statistical classification method that uses knowledge of probability and statistics for classification. The principle is to use the Bayesian formula to calculate the posterior probability of the sample according to the prior probability of the sample and select the class label with the largest posterior probability as the final sample. Presently, there are mainly four kinds of Bayesian classifiers that have been studied more, namely, Naive Bayes, TAN, BAN, and GBN. We mainly introduce the Naive Bayes classification.

*I*. *Naive Bayes Algorithm*. Suppose an n-dimensional feature vector is used to describe a sample with *n* attribute values, namely, *X*{*x*_1_, *x*_2_,…, *x*_*n*_}, assuming that there are *m* class labels, denoted by *C*_1_, *C*_2_,…, *C*_*m*_. For a sample, *X* with an unknown class label, if Naive Bayes classification is used to assign *X* to class *C*_*i*_, the following equation holds:

(1) $$\begin{array}{c} P\left(C_{i}X\right)>P\left(C_{j}X\right),\;1\leq j\leq m,\;j\neq i. \end{array}$$

According to Bayes' theorem,

(2) $$\begin{array}{c} P\left(C_{i}X\right)=\frac{P\left(X|C_{i}\right)P\left(C_{i}\right)}{P\left(X\right)}. \end{array}$$

Because *P*(*X*) is a constant for all classes, maximizing the posterior probability *P*(*C*_*i*_*X*) can be expressed as maximizing the prior probability *P*(*X|C*_*i*_)*P*(*C*_*i*_); if the training set has more Attributes and tuples, the cost of calculating *P*(*X|C*_*i*_) will be very large, so in general, it is assumed that the values of each attribute are independent of each other, so

(3) $$\begin{array}{c} P\left(XC_{i}\right)=\prod_{i}^{n}P\left(X_{i}|C_{i}\right). \end{array}$$

The prior probability *P*(*X*_1_*C*_*i*_), *P*(*X*_2_*C*_*i*_),…, *P*(*X*_*n*_*|C*_*i*_) can be obtained from the training dataset.

Therefore, for a sample *X* of an unknown class mark, the probability *P*(*XC*_*i*_)*P*(*C*_*i*_) that *X* belongs to each class mark Ci can be calculated first, and then the class mark with the highest probability is selected as its final class mark, that is, the classification result.

The article "Nursing Diagnosis of Urology Operating Room Based on New Association Classification Algorithm" was retracted in 2023. Reasons: signs of a paper mill; compromised peer review; unreliable results or conclusions.

The premise of using the Naïve Bayes classification algorithm is that the attributes are independent of each other. Only when the dataset satisfies the independence assumption, the classification accuracy will be higher, otherwise it will be lower. In addition, the algorithm does not output classification rules.

The Naïve Bayes classification algorithm can be applied to situations with large datasets, and is relatively simple, with high classification accuracy and fast speed.

#### 3.1.4. BP Artificial Neural Network

(i) Basic Concepts
    Artificial neural network is a model that simulates the mechanism of biological neurons. In organisms, a neuron network is a loosely interconnected network composed of a huge number of neurons. The stimulus (input) coming in from the outside world produces various responses (outputs) through the transmission and interaction between neurons, which embodies various functions. The strength of the connection between neurons will change under different inputs, so as to learn the correct response under different input situations.
    To mimic this mechanism, artificial neural networks are also composed of a group of neurons and the connections between them. The neuron responds according to its input (determined by the excitation function), and the strength of the connection (called the weight) is continuously adjusted with the input until it responds correctly to all inputs. Artificial neural networks have a variety of connection modes to form a multi-purpose network. The most commonly used one is the feedforward neural network, which is a hierarchical artificial neural network, mainly used for classification and prediction.
    A typical feedforward neural network consists of an input layer, an output layer, and several intermediate layers (also called hidden layers). Each layer is composed of several neurons (also called nodes). The nodes between the layers are fully connected. The nodes in the layer are not connected.
    BP artificial neural network (back propagation, error backpropagation network) is a multi-layer feedforward neural network that uses a minimum mean square error learning method. It is a learning process supervised by a tutor and is currently the most widely used neural network.
(ii) Basic Idea of BP Algorithm
    The learning process of BP artificial neural network is divided into two steps: signal forward propagation and error back propagation.
(iii) Forward Propagation of the Signal
    The input samples start from the input layer, are processed layer by layer by the hidden unit, and after passing through all the hidden layers, they are passed to the output layer to produce output results. In this process, the state of each layer of neurons only affects the state of the next layer of neurons, and the connection weight of the network is fixed. In the output layer, the actual output and the expected output are compared. If the two are not equal, then the process of back propagation of the error is turned to.
(iv) Back Propagation of Errors
    The difference between the actual output and the expected output is the error signal. The error signal is transmitted back according to the previous forward propagation path, and the weight coefficient of each neuron in each hidden layer is modified to ensure that the error signal trend is the smallest. The process of using the forward propagation of the signal and the backward propagation of the error to adjust the connection weights of each layer is repeated. The learning and training process of the neural network is a process of continuously adjusting the weights. The process will not stop until the output error of the network reaches an acceptable level or reaches the maximum number of learning set at the beginning.

The article "Nursing Diagnosis of Urology Operating Room Based on New Association Classification Algorithm" was retracted in 2023. Reasons: signs of a paper mill; compromised peer review; unreliable results or conclusions.

#### 3.1.5. Classification Based on Association Rules

In 1993, Agrawal first proposed the concept of association rule mining, and it is currently one of the hotspots in the field of data mining. The initial purpose of association rule mining is to discover consumer shopping behavior rules from the supermarket transaction database. Association rules describe a hidden relationship between two or more attributes.

The basic task of mining association rules is to first dig out strong association rules in large databases by specifying minimum support and minimum confidence by users. The problem of association rule mining can be divided into two subproblems: one is to mine the frequent item set, and the other is to generate association rules that users are interested in based on the frequent item set mined.

(i) Mining Frequent Item Set
    Use the specified minimum support min sup to find all frequent item sets, that is, all item sets full of support > min sup.
(ii) Generate Association Rules
    Use frequent item sets to generate association rules whose confidence is greater than a predetermined minimum confidence threshold. After the frequent item sets are determined, the corresponding association rules can be easily derived. Therefore, the core problem of most mining algorithms is how to efficiently calculate frequent item sets. The first sub-problem has become the focus of research on association rule algorithms in recent years. Many classic frequent item set mining algorithms have also been proposed.
    The Apriori algorithm was proposed by R. Agrawal and R. Srikant in 1994 which is used to mine all frequent item sets. It uses the breadth-first iterative search method to first find 1-frequent item set F1which is used to find 2-frequent item set F2. F2 uses it to find and then loops until the frequent k-items set cannot be found. Finally, the database is scanned once to find each *F*_k_.

The article "Nursing Diagnosis of Urology Operating Room Based on New Association Classification Algorithm" was retracted in 2023. Reasons: signs of a paper mill; compromised peer review; unreliable results or conclusions.

### 3.2. Research on the Urological Diagnosis Based on the New ACCF

This paper proposes a new associative classification based on closed frequent item set (ACCF) algorithm. The main contributions of this are as follows:

- A new method for constructing a classifier with higher accuracy is proposed. ACCF produced a smaller number of candidate rule sets with higher quality. Experimental results show that the average classification accuracy of the classifier constructed by ACCF is higher than that of CBA. Compared with the classification algorithms introduced in Section 3, its classification accuracy rate on the urology dataset is also the highest, which meets the requirements of the urology clinical decision support system for the core classification algorithm.
- Solve some key problems in the actual classification system. When the dataset contains a large number of rules, the use of CBA and CMAR algorithms, whether it is rule generation or rule selection, is very time-consuming. In practice, if there is no rule restriction, some datasets cannot even be ruled mining at all. ACCF can produce a rule set with a small quantity, high quality and no redundancy.
- For association classification, a new framework based on frequent closed item set is proposed.

First, define a sample database and express it in two forms, horizontal and vertical (as shown in Table 1):

Let *I*={*i*_1_, *i*_2_,…, *i*_*m*_} be a set of items (item set), *D*={*t*_1_, *t*_2_,…, *t*_*m*_} be a set of data transactions, use 〈tid, *X*〉 to represent each transaction, tid is its identifier, and *X* is its corresponding item.

#### 3.2.1. Item Set and Identification Set

If the set X⊆ I, then X is an item set. If Y⊆T, then Y is a tidset. The set of all tidsets is identified as T. The set consisting of k(k > 0) items is called the k-item set. For simplicity, the item set {*A*, *C*, *W*} is abbreviated as ACW, and the identity set {2, 4, 5} is abbreviated as 245. For an item set X, its corresponding identification set is represented as *t*(*X*) , that is, the set of identifications of all transactions that contain X. For an identity set Y, its corresponding item set is denoted as *i*(*Y*), that is, the set of items whose identities of all transactions are in Y. Denote it as *t*(*X*)=*I*_*x*∈*X*_*t*(*x*),  *i*(*Y*)=*I*_*y*∈*Y*_*i*(*y*). For example, in Table 1, *t*(*ACW*)=*t*(*A*)∩*t*(*C*)∩*t*(*W*)=1345∩123456∩12345∩1345,  *i*(12)=*i*(1)∩*i*(2)=*ACTW*∩*C*  *DW*  ∩*CW*.

The article "Nursing Diagnosis of Urology Operating Room Based on New Association Classification Algorithm" was retracted in 2023. Reasons: signs of a paper mill; compromised peer review; unreliable results or conclusions.

#### 3.2.2. Closed Item Set

Let *c* : *p*(*I*)⟶*p*(*i*) be the closed operator, and define *c*(*X*)=*i*(*t*(*X*)), *X* ∈ *I*. The frequent item set *X* is closed if and only if *c*(*X*)=*X*.

#### 3.2.3. Frequent Closed Item Set

The support of item set *X* is the number of transactions that contain *X*, denoted as sup(*X*), namely, sup(*X*)=|*t*(*X*)| . The item set that meets the support degree greater than or equal to the given minimum support threshold (mins up) is called the frequent item set, namely, sup(*X*) ≥ min sup. The so-called frequent closed item sets are those whose support degree is greater than the support degree of any superset.

## 4. A New Association Algorithm Based on Frequent Closed Item Sets

### 4.1. The Production Process

Association classification algorithms usually include two stages, one is rule generation and classifier establishment stage, and the other is how to use the classifier to perform classification. ACCF also includes the above two stages. The steps for ACCF to generate class association rules are as follows:

1. Generate candidate association rules. ACCF uses the CHARM algorithm to generate all CFIs and corresponding identification sets of the training dataset. The sup(R) and conf(R) of CARs can be calculated by the intersection of the two identification sets. ACCF only generates minimal association rules, avoiding a large number of redundant association rules, which is much less than the number of rules generated by general classification algorithms (such as CBA).
2. ACCF only selects rules whose support and confidence are both greater than the corresponding threshold, and then selects only a part of the rules as the rules of the classifier by avoiding redundant rules and pruning rules. The classifier at this time contains all frequent and high-quality rules.

In the classification stage, the following problems are mainly solved: given a data object, how to match the most effective rules when classifying a new instance.

This section introduces the method of generating candidate classification rules and the basic principle that ACCF only generates minimum association rules.  Figure 2 shows a closed set represented by an item set identification set search tree (IT-tree). The following example illustrates the main idea of ACCF mining rules.

**Example 1 .**

(Mining Association Rules). Let *T* be the training dataset, as shown in Table 2.

For the dataset shown in Table 2, IT-tree structure obtained by the CHARM algorithm is as follows:

Figure 2 shows the frequent closed item set and their corresponding tids obtained by mining the CHARM algorithm when we regard the class labels as general items. The rules in ACCF are defined as: <rule, support, confidence>. Assuming that the minimum support is 1%, ACCF has 17 candidate association rules obtained from the dataset in Table 2.

The article "Nursing Diagnosis of Urology Operating Room Based on New Association Classification Algorithm" was retracted in 2023. Reasons: signs of a paper mill; compromised peer review; unreliable results or conclusions.

Using traditional association classification algorithms, such as CBA, the number of candidate rules generated is 81. ACCF greatly reduces the number of redundant association rules.

#### 4.1.1. ACCF Only Generates Minimal Association Rules

When ACCF generates candidate association rules, compared with traditional association classification algorithms such as CBA, it only generates minimum association rules, which can eliminate redundant association rules.

For a frequent item set S of size *L*, since S has 2L subsets, subtracting S itself and the empty set that cannot be the antecedent of the association rule, 2L-2 association rules may be generated. Therefore, the complexity of generating association rules for frequent item set is O(N2k), where N represents the number of frequent item set, and *k* represents the length of the longest frequent item set. However, the support and confidence of some association rules extracted from frequent item sets are the same, and they do not provide new useful information, that is, there are a lot of redundant association rules. The traditional association classification algorithm does not deal with these redundant rules.

We call the rules that cannot be deduced from other rules and whose support and confidence are the same as those of other association rules as minimum association rules. As long as we find all the minimum association rules, we can get all the association rules by adding the relevant item set to the antecedent or subsequent parts of the minimum association rule.

After the ACCF classification model is constructed, the classification model needs to be evaluated, that is, in the classification stage, we use the test dataset to evaluate the accuracy of ACCF classification. Generally, the overhead of the classification stage is much lower than that of the rule set generation stage.

The concept that the rules in the ACCF match the objects in the test dataset: if a data object obj matches the pattern *P*=*a*_*i*1_,…, *a*_*ij*_,…, *a*_*ik*_, then 1 ≤ *j* ≤ *k*. The value on each Aij is aij. This matching method is the same as the association classification algorithm based on general frequent items. For an object obj to be classified, if a classification rule *x*˗*c* matches the object to be classified, it satisfies the following principles:

1. Match experience association rules. According to doctors' accumulated experience in long-term clinical practice, some empirical association rules are formed;
2. If obj contains all the attribute values in *x*, such as obj=*C*  *DT*  *W*, then the rule *C*  *DT*  ˗*N*  is the matching classification rule, and the class label of the object obj is *N*;
3. If the object obj cannot find the rule antecedents that it can completely contain in the classification rules, then find the rule whose intersection is not zero from the rules. For example, obj=*C*  *D*, the rule *C*  *DT*  ˗*N*  is also the matching classification rule;
4. If the above two principles still cannot find a matching rule, the default class will be matched. Among them, principles 2 and 4 are the matching methods of the CBA algorithm, and principles 1 and 3 are the matching methods defined by us. After adding principles 1 and 3, the accuracy of classification can be effectively improved.

The article "Nursing Diagnosis of Urology Operating Room Based on New Association Classification Algorithm" was retracted in 2023. Reasons: signs of a paper mill; compromised peer review; unreliable results or conclusions.

### 4.2. ACCF Experiment on UCI Dataset

#### 4.2.1. Experimental Data

In order to test the performance of the ACCF algorithm proposed in this article, this article selects the standard data in the data mining field to compare the performance of different algorithms. 18 datasets include Austra, Auto, breast, Cleve, Crx, diabetes, glass, heart, hepatitis, Horse, Iris, labor, led7, pima, tic, Vehicle, Wave, and wine.  Figure 3, Figure 4, and Figure 5 give detailed information on the 18 datasets.

#### 4.2.2. Verification Method

Using 10-fold cross-validation for 18 UCI datasets, each dataset is divided into 10 points, S_1_, S_2_, ..., S_10_; training and testing are performed 10 times, and in the i-th iteration, *S*_*i*_ is used as the test set, and the rest as the training set. The number of class association rules and the number of classifier rules are the average of 10 iterations. The classification accuracy is the average of the ratio of the number of correct classifications to the total number of samples.

#### 4.2.3. Benchmark Method

Since the CBA algorithm is a typical representative of the association classification algorithm based on frequent item set, in order to analyze the effectiveness of the algorithm proposed in this paper, only ACCF is used in this experiment to compare with it. By running the two on 18 datasets, respectively, to test their classification accuracy and the number of candidate association rules, it demonstrates the effectiveness of the proposed algorithm in this paper.

#### 4.2.4. Experimental Results

The experimental parameters are set as follows: minsup is 1%, minconf is 50%, the dataset coverage threshold is 4, and the rule number threshold is 80000.

The article "Nursing Diagnosis of Urology Operating Room Based on New Association Classification Algorithm" was retracted in 2023. Reasons: signs of a paper mill; compromised peer review; unreliable results or conclusions.

Table 3, Table 4, Figure 6, and Figure 7 compare the ACCF algorithm and the CBA algorithm in terms of the number of association rules and classification accuracy, respectively. The experimental results show that ACCF is more efficient in the number of CARs generated, and the size and accuracy of the classifier.

The first column of Tables 3 and 4 is the name of the 18 UCI datasets. The dataset marked with ∗ indicates that the rules need to be restricted when the CBA algorithm is used to construct the classifier. The restricted rules include CARs and support and confidence. The degree is less than a predetermined threshold. The last two columns of Table 3 list the number of CARs generated by the two algorithms. For each experimental dataset, the number of candidate CARs generated by the ACCF algorithm is much less than that of the CBA algorithm, which is on average 1/5 of the latter. The second and third columns of Tables 3 and 4 give the size of the classifier in terms of the number of rules. ACCF produced a smaller classifier in most of the datasets. The last two columns are the corresponding average classification accuracy, which increased from 83.4% of CBA to 86.1% of ACCF. Specifically, ACCF showed better classification accuracy in 14 of 18 datasets. This verifies that the quality of the rules generated by frequent closed item sets is higher and the classification accuracy is improved.

### 4.3. ACCF Experiment on Urology Disease Data Set

#### 4.3.1. Experimental Data

The urology dataset used in this experiment has been mentioned in the previous article, so I will not repeat it here.

#### 4.3.2. Verification Method

A 10-fold cross-validation is also used for the urology dataset.

#### 4.3.3. Benchmark Method

Compared with several traditional classification algorithms, namely, ID3, C4.5, Naive Bayes, BP neural network, and CBA algorithm introduced in Section 3, the classification accuracy is compared.

#### 4.3.4. Experimental Results

The experimental parameters of ACCF and CBA are set as follows: minsup is 1%, minconf is 50%.

On the urological disease dataset, the experimental results in Table 5 show that compared with CBA, ACCF greatly reduces the number of candidate association rules, from 9308 in CBA to 2228 in ACCF, and the number of classifier rules is changed from CBA. The number of ACCF articles were reduced from 49 to 22. The experimental results in Figure 8 show that, compared with the traditional data mining classification algorithm introduced in Section 3, ACCF has the highest classification accuracy rate of 91.7%, which meets the requirements of the urology clinical decision support system for the core classification algorithm.

The article "Nursing Diagnosis of Urology Operating Room Based on New Association Classification Algorithm" was retracted in 2023. Reasons: signs of a paper mill; compromised peer review; unreliable results or conclusions.

## 5. Conclusion

In recent years, medical engineering has developed rapidly, and a large amount of medical data are recorded in detail through measuring instruments, which has led to a massive increase in medical-related data. In such a massive database, various data mining methods and techniques are used to discover and summarize the clinical manifestations, development rules, and interrelationships of various diseases, and compare the efficacy of various diagnosis and treatment programs. This is pertinent even for the diagnosis and treatment of diseases. Medical research is very valuable and meaningful.

This paper first reviews the diagnosis of urological diseases based on traditional data mining classification methods, and then proposes a new association classification algorithm based on the frequent closed item set, ACCF. The ACCF algorithm is based on frequent closed item sets, and all frequent item sets can be obtained according to frequent closed item sets. The class association rules obtained by the frequent closed item set can get all the rules. Combined with the characteristics of urological disease data, the ACCF algorithm has also been improved in rule pruning and matching methods. Experiments on the 18 datasets and urological disease datasets in the UCI database show that ACCF can mine high-quality rules without any loss of information. This not only greatly reduces the number of candidate association rules but also provides a classification with a high accuracy rate. It is also higher than the representative traditional association classification algorithm—CBA algorithm. In the diagnosis of urological disease sets, ACCF also showed the highest classification accuracy rate compared with other traditional classification algorithms introduced in this article.

There are a large number of excellent other classification algorithms in data mining, which can be used to construct the classifier of the urology clinical decision support system; therefore, in future, we can use other algorithms to continue the research work of this article. For example, due to the limited samples in the experiment, a support vector machine algorithm suitable for small sample learning can be used. Follow-up work can also be carried out in other medical fields based on the ideas and algorithms in this article for further research.

## Figures and Tables

**Figure 1:** Urology surgery nursing.

**Figure 2:** Mining result of CHARM algorithm.

**Figure 3:** Comparison of the number of attributes on different datasets.

**Figure 4:** Comparison of the number of samples on different datasets.

**Figure 5:** Comparison of the number of classes on different datasets.

The article "Nursing Diagnosis of Urology Operating Room Based on New Association Classification Algorithm" was retracted in 2023. Reasons: signs of a paper mill; compromised peer review; unreliable results or conclusions.

**Figure 6:** Accuracy of the CBA algorithm.

**Figure 7:** Accuracy of the ACCF algorithm.

**Figure 8:** Comparison of Classification Accuracy between ACCF and others.

**Table 1:** Sample dataset.

Database			
Transaction	Items	Transaction	Items
1	ACTW	A	1345
2	CDW	C	123456
3	ACTW	D	2456
4	ACDW	T	1356
5	ACDTW	W	12345
6	CDT	—	—

**Table 2:** Training dataset.

Tid	Items	Class label
1	ACTW	Y
2	CDW	Y
3	ACTW	Y
4	ACDW	N
5	ACDTW	N
6	CDT	N

**Table 3:** Count comparison of CARs.

Dataset	CBA/CARs	ACCF/CARs
Austra	65082	8594
Auto	50237	1079
Breast^*∗*^	2832	4443
Cleve	48855	12711
Crx	42878	9669
Diabete^*∗*^	3316	586.5
Glass^*∗*^	4235	338.7
Heart^*∗*^	52310	5268
Hepatitis	42878	8563
Horse	62746	12746
Iris^*∗*^	73	63
Labor^*∗*^	5566	580.4
led7^*∗*^	465	1276
Pima^*∗*^	823	586
Tic^*∗*^	6487	6284
Vehicle	56954	7898
Wave^*∗*^	9700	688
Wine^*∗*^	38071	12558
Average	27456.2	5217.6

**Table 4:** Comparison of dataset rules.

Dataset	CBA rules	ACCF rules
Austra	172	126.7
Auto	63	52.5
Breast^*∗*^	64	58.1
Cleve	92	80.6
Crx	179	167.7
Diabete^*∗*^	66	56.1
Glass^*∗*^	33	22.7
Heart^*∗*^	53.2	51
Hepatitis	43	29.9
Horse	123	90.2
Iris^*∗*^	10	6.7
Labor^*∗*^	18	12.2
led7^*∗*^	46	64.5
Pima^*∗*^	66	56.7
Tic^*∗*^	32	103.1
Vehicle	148	65.6
Wave^*∗*^	661	491.1
Wine^*∗*^	11	8.8
Average	104.5	82.1

**Table 5:** Number comparison of CARs between ACCF and CBA.

Algorithm	Number of CARs	Number of classifiers
CBA	9308	49
ACCF	2228	22

## Data Availability

The datasets used are available from the corresponding author on reasonable request.
